# Localized and Generalized Skin Adverse Drug Reactions to Nadroparin Calcium Injection in 6 Cases of Pregnant Women

**DOI:** 10.1155/2022/5622482

**Published:** 2022-04-15

**Authors:** Ting Chen, Liling Lan, Wenwen Sun, Jia Yu, Baozhen Lu, Lijie Chen, Liwei Sun, Zhendong Yu, Bo Wu, Ying Xiong

**Affiliations:** ^1^Department of Dermatology, Affiliated Shenzhen Maternity & Child Healthcare Hospital, Southern Medical University, Shenzhen 518000, China; ^2^Department of Reproductive Immunology, Affiliated Shenzhen Maternity & Child Healthcare Hospital, Southern Medical University, Shenzhen 518000, China; ^3^Central Laboratory, Peking University Shenzhen Hospital, Shenzhen 518000, China

## Abstract

**Background:**

Despite the increasing number of skin adverse drug reactions caused by nadroparin calcium have been reported, mostly, little is known regarding of their details of clinical characteristics, especially for generalized skin adverse drug reactions. We sought to evaluate localized and generalized characteristics of the skin adverse drug reaction to nadroparin calcium injection in pregnant women.

**Methods:**

A retrospective study was conducted on 6 pregnant women, who experienced localized and generalized skin adverse drug reactions during long-term nadroparin calcium injection. The patients' clinical and imaging information were retrieved from medical records. The skin prick test, patch test, and intradermal test were performed after they stopped lactation. Causality assessment of suspected adverse drug reactions was performed on these cases.

**Results:**

The average total dose of nadroparin calcium injection in the 6 cases was 64.17 ± 22.66. Localized skin adverse drug reaction, manifested as erythema at the injection point, appeared after 47.5 ± 17.4 days of subcutaneous injection of nadroparin calcium. Generalized urticaria-like lesions, progressing from the injection site on the abdomen, appeared in 5.17 ± 3.60 days after the first appearance of localized reaction, while laboratory test results revealed essential peripheral blood eosinophilia. All rashes in the 6 cases subsided in 2–5 weeks after drug withdrawal. After delivery, 5 of 6 cases received complete skin tests to evaluate drug hypersensitivity. Results presented positive in the intradermal test within 7 days. Both the skin prick test and skin patch test were negative. Localized skin reactions and generalized urticaria-like adverse drug reactions were considered as definitely and probably caused by nadroparin calcium injection, respectively.

**Conclusion:**

Subcutaneous injection of nadroparin calcium in pregnant women appears to be at risk of localized and generalized urticaria-like adverse drug reaction. It is important to follow up the pregnant woman during nadroparin calcium injection for evaluating adverse drug reactions. Timely detection of symptoms is pivotal in early diagnosis and treatment of adverse drug reactions.

## 1. Introduction

Nadroparin calcium is one kind of low-molecular-weight heparins, obtained by the depolymerization of unfractionated heparin. Nadroparin calcium has a strong antifactor Xa activity. It is a classic anticoagulant. Due to the high safety and bioavailability, nadroparin calcium is majorly used to treat and prevent thrombotic diseases [1]. Studies have demonstrated that low-molecular-weight heparins can improve the microcirculation of the uterus and placenta in pregnant women with recurrent miscarriage, thereby reducing the risk of miscarriage [2]. Therefore, in recent years, low-molecular-weight heparins are widely used in the department of obstetrics and gynecology, as well as in the department of reproductive medicine [2]. However, with the widespread clinical usage, adverse drug reactions caused by such drugs have been reported from time to time [3–5]. In this study, we retrospectively reviewed the clinical data of pregnant women who underwent nadroparin calcium injection and experienced localized and generalized skin adverse drug reactions. We analyzed and summarized characteristics and outcomes of these cases, aiming to improve clinicians' understanding of this issue.

## 2. Materials and Methods

### 2.1. Materials

Clinical data of pregnant women with recurrent miscarriage were retrospectively collected. These women were admitted in the Department of Dermatology at the Affiliated Shenzhen Maternity and Child Healthcare Hospital, Southern Medical University, from June 2019 to May 2020. Only the pregnant women experiencing localized and generalized skin adverse drug reactions after received nadroparin calcium (product name: Subilin) would be evaluated. Ethical approval was obtained from the Ethics Committee of Affiliated Shenzhen Maternity and Child Healthcare Hospital, Southern Medical University.

### 2.2. Data Collection

The data encompassed age, indication for nadroparin calcium application, combined medication, incubation period between beginning of nadroparin calcium to onset of symptom, and total injection dose. 2 main clinical complaints were recorded: (a) localized skin adverse drug reaction (also known as injection site reaction) and (b) generalized skin adverse drug reaction. We additionally recorded the characteristics of generalized skin reaction and the interval between the onset of localized and generalized skin adverse drug reaction.

### 2.3. Patient Screening

To explore the reason and exclude other pathologies, some routine blood tests and liver function tests were performed in these pregnant women. Treatment information and the follow-up information of the patients were retrieved from medical records and the telephone, respectively.

Skin tests are of high significance for the evaluation of drug hypersensitivity reactions. However, it is not ethical to perform the skin test during pregnancy and lactation; we invited the patient to receive the skin test after they stopped lactation.

### 2.4. Skin Stimulation Test

All but 1 patient in the study performed 3 challenge tests (skin prick test, patch test, and intradermal test). The selected contraction and method to the skin test was referenced by the ENDA/EAACI Drug Allergy Interest Group [6]. Nadroparin calcium's concentrations in 3 skin tests were, respectively, undiluted (prick), 1/10 diluted (intradermal), and undiluted (patch), while the control group only received saline solution. Patch tests were occluded for 48 hours using 8 mm Finn Chambers® on Scanpor® tape (Smart Practice, America), and readings were performed according to ICDRG criteria. The case with the negative patch test in 7-day follow-up would accept the skin prick test and intradermal test.

### 2.5. Causal Relationship Assessment

According to Uppsala Monitoring Centre of WTO's recommendation [7], causality assessment of suspected adverse drug reactions was performed on these cases.

## 3. Results

### 3.1. General Characteristics

Clinical data of 6 pregnant women were collected and reviewed. The underlying disease of these pregnant women was recurrent miscarriage. According to the doctor's order in the Department of Obstetrics and Gynecology or Department of Reproductive Medicine, they underwent a long course of subcutaneous nadroparin calcium injection. The injection site was the abdomen for all individuals. The injection frequency was once every two days, once per day, or twice per day. The average total dose was 64.17 ± 22.66 (Table 1).

### 3.2. Symptoms and Time of Appearance of Skin Adverse Drug Reactions

The initial symptom of all individuals appeared at the injection point, manifested as erythema accompanied with itching (Figure 1). As given in Table 1, the average incubation period (duration between the first injection and the initial symptom appearance) was 47.5 ± 17.4 days. On average, the erythema at each injection point gradually subsided in 3.33 ± 1.21 days. After the appearance of the initial symptom, the individual changed the injection point. On average, delayed reactions reappeared in 6.67 ± 3.08 hours. Generalized skin reactions appeared in 5.17 ± 3.60 days after the initial symptom. All of the 6 cases experienced severe skin itching. Five individuals exhibited urticarias progressed from the injection site on the abdomen to other body parts, including the trunk, limbs, eyelids, and fingers. One individual only experienced skin itching with no wheal. However, dermatographism could be seen (Table 1).

### 3.3. Auxiliary Examinations

All 6 individuals underwent routine blood tests and liver function tests when they received heparin treatment regularly. At the time of referral to dermatologist, they were again be checked with routine blood tests and liver function. Results indicated that for all individuals, platelets were always in the normal range, while the liver function did not show any abnormality. Therefore, heparin-induced thrombocytopenia and drug-induced liver injury could be ruled out. However, when they presented to dermatology, the average absolute eosinophils count among the 6 individuals was (0.55 ± 0.34) × 10^9^/L, while the normal range was only 0.02–0.05 × 10^9^/L.

### 3.4. Treatments and Outcomes

After the appearance of localized and generalized skin adverse drug reactions, all 6 individuals stopped nadroparin calcium injection. One individual replaced nadroparin calcium with fondaparinux and another individual replaced with enoxaparin, while the other 4 individuals stopped taking any anticoagulant therapy after the drug withdrawal. Three individuals with severe symptoms underwent topical corticosteroids therapy to treat localized adverse drug reactions and took loratadine and chlorpheniramine to treat generalized adverse drug reactions. Adverse drug reactions at the injection point and urticarias subsided in 2–5 weeks in all individuals.

### 3.5. Skin Test

When the cases stopped lactation, they received our invitation to perform the skin test for confirmation of drug hypersensitivity reaction. They accepted the invitation except 1 case. The results showed the patch test was negative, while the prick test was also negative. However, with the 7-day follow-up, the intradermal test of 5 other cases indicated positive result, presented in injection sites of culprit heparin, but the negative control with saline showed negative result.

### 3.6. Causality Assessment of Suspected Adverse Drug

According to the World Health Organization-Uppsala Monitoring Centre (WHO-UMC) causality categories, causality assessment of suspected adverse drug was performed.

#### 3.6.1. Time Sequence of Medication and Adverse Drug Reactions

All individuals were undergoing nadroparin calcium injection before experiencing localized skin adverse drug reactions. The average incubation period was 47.5 ± 17.4 days, which was close to the 50 (5–185) days incubation period reported in previous studies [8].

#### 3.6.2. Outcomes after Drug Withdrawal

All individuals stopped nadroparin calcium injection after the appearance of localized and generalized symptoms. Both localized and generalized skin adverse drug reactions were obviously improved after the drug withdrawal.

#### 3.6.3. Reappearance of Adverse Drug Reactions

Localized reactions appeared in all cases after changing the injection point. However, currently, we have not observed the reappearance of generalized skin adverse drug reactions of reinjection after drug withdrawal. Skin tests during pregnancy and lactation do not meet ethical requirements. Therefore, skin tests including prick, patch, and intracutaneous tests were performed after stopping lactation. Except 1 subject who declined the intradermal test, all other 5 subjects received a positive result in intradermal tests within 7-day follow-up, which showed urticaria-like in the injection site, but both prick and patch tests were negative.

#### 3.6.4. in Accordance with Known Type of Adverse Drug Reaction

The drug instruction describes adverse drug reactions including urticarial, erythema, and itching, which belong to rare adverse drug reactions. It reported urticarial lesion at the injection site after 8–29 days of subcutaneous injection of low-molecular-weight heparins [9].

#### 3.6.5. Exclusion of Other Primary Diseases and Confounding Factors

Although most patients with recurrent miscarriage combine other drugs, such as dydrogesterone, with heparin together in the treatment, by checking the medical history and communicating with the individual, we confirmed that all of the 6 individuals had used dydrogesterone and/or other drugs multiple times, but never experienced any allergic reaction. After the appearance of generalized skin adverse drug reactions, all individuals only stopped the nadroparin calcium injection, but still continued using other drugs. Moreover, both localized reactions and generalized urticaria-like reactions arised from the injection site around the abdomen, suggesting that the tight relationship between rashes and nadroparin calcium.

In summary, we consider localized reactions at the injection point as definitely caused by the nadroparin calcium injection and generalized urticaria-like reactions as probably caused by the nadroparin calcium injection.

## 4. Discussion

Skin damage is the most common adverse drug reaction of heparin subcutaneous treatment [10, 11]. Heparin-induced skin lesions can manifest in many forms, such as immediate hypersensitivity, skin necrosis caused by immune-mediated thrombocytopenia, and delayed hypersensitivity. It can also cause rare cases, such as acute generalized exanthematous pustulosis [12].

Among various types of skin reactions, immediate hypersensitivity reactions may be caused by chondroitin sulfate of the incomplete heparin purification. Along with the improvement of production technologies, the incidence of immediate hypersensitivity is gradually decreasing [12]. Immune-mediated thrombocytopenia is the most serious skin reaction caused by heparin. In this case, the formation of the heparin-platelet factor 4-IgG antibody leads to the destruction and reduction of platelets. It may also accompany the formation of arterial and/or venous thrombosis. The mortality rate can reach as high as 20–30% [13]. However, the incidence is relatively low, ranging from 0.1% to 5%. The delayed hypersensitivity at the injection point is the most common type of heparin-induced skin damage. It usually manifest as erythema at and around the injection point. The incidence in the general population can reach 10.3% [14]. In pregnant women, the incidence of heparin-induced skin adverse drug reactions is among 19.8–39.9%, which is 2–4 folds higher than nonpregnant females. Therefore, pregnancy is considered as a high-risk factor for delayed allergic reactions induced by heparin [8]. Although, high-risk factors for delayed hypersensitivity reactions also include gender, obesity, treatment time, or dosage, the choice of anticoagulants seems to be more likely to induce hypersensitivity reactions than any other identified risk factors [4, 8]. Nadroparin calcium has the highest incidence to cause skin lesions (approximately 65% at 100 days), which is much higher than dalteparin sodium and enoxaparin. Scholars speculate that the hypersensitivity of nadroparin calcium may be related to its special antigenic determinants [8].

Localized reactions at the injection point reported in this study is consistent with the previous studies. We further elaborated on the time of the appearance and disappearance of reactions at the injection point. After the appearance of the initial symptom, it only took less than 10 hours for reactions appearing at new injection points. These localized reactions can gradually subside in 5 days. More importantly, we observed that all 6 individuals exhibited generalized urticaria-like rash accompanied with severe itching in 1–7 days after the appearance of localized reactions. In addition, several individuals' blood routines suggested increased eosinophils count. This alteration has never been discovered in the earlier obstetric examinations, indicating that the increase of eosinophils count was caused by nadroparin calcium. In the past, there were relatively few reports about heparin-induced generalized skin adverse drug reactions. The first related case was reported in 2003 about generalized erythema caused by enoxaparin [15]. In 2010, a study reported appearances of generalized erythema after 40 hours of low-molecular-weight heparin usage [16]. Later, there were some studies which discovered that generalized eczematous reactions could be induced by severe localized reactions at the inject point [4, 14, 17]. However, in previous literature, we did not find any report about generalized urticaria-like reactions appeared after 1-2 months of heparin usage. We speculated that this phenomenon might be explained by the following reasons. (1) As mentioned above, with the extension of time or the increasing doses, the probability of skin adverse drug reaction to nadroparin calcium may increase. All the 6 cases received medicine over 47.5 ± 17.4 days, and this may be an unreported adverse drug reaction of long-term subcutaneous injection of nadroparin calcium. (2) Adverse drug reaction is affected by many factors, including genetic and immunological factors. Therefore, we cannot exclude the possibility that races, populations, or gestation are involved in the pathogenesis of skin adverse drug reaction.

Regarding the pathogenesis of generalized urticaria-like reactions, we reviewed the literature and found it is common of eosinophils count increase during long-term subcutaneous heparin treatment [16, 18, 19]. The continuous antigen presentation activates CD4^+^ T cells, which leads to the recruitment and activation of eosinophils. Increased eosinophils release tissue-damaging proteins and produce many other proinflammatory and immunomodulatory molecules. This is considered as one of the pathogeneses of urticaria [20]. We hypothesize that this is also the pathogenesis of urticaria-like reactions induced by long-term subcutaneous injection of nadroparin calcium.

Since adverse drug reactions are one of the common causes for poor adherence to treatment, how to avoid its adverse reactions is the key to improve the effect for recurrent miscarriages. Regrettably, more researches are needed to elucidate the pathogenesis of adverse drug reactions. Nevertheless, early detection of skin adverse drug reaction to heparin is important to alleviate suffering and improve life quality. When localized or generalized rash appears during treatment with heparin anticoagulation, physicians need to be alerted to the development of skin adverse drug reaction to heparin, especially in patients under long-term treatment. Once skin adverse drug reaction is suspected, heparin is recommended to be stopped. Our study found that the rash subsided in 2–5 weeks after stopping nadroparin calcium injection. During this period, based on the individual's needs and the severity of symptoms, oral and/or topical drugs can be used to relieve itch. For those individuals who still need anticoagulant therapy, we need to select effective alternative anticoagulants. It has been reported that 33–73% individuals may develop cross-allergic reactions between different low-molecular-weight heparins [12]. In this study, one individual replaced nadroparin calcium with enoxaparin. No cross-allergic reaction was discovered. In addition, fondaparinux is a chemically synthesized sulfated pentasaccharide, which can specifically inhibit coagulation factor Xa. It has been demonstrated in several clinical studies that fondaparinux can be well tolerated in individuals with allergies to heparin. It can be used as the primary alternation in pregnant women with heparin allergies [4].

## 5. Conclusion

Nadroparin calcium is a classic drug for the treatment of recurrent miscarriage. However, skin adverse drug reactions to nadroparin calcium cannot be ignored, which may cause new health problems. Long-term injection of nadroparin calcium may cause localized and generalized skin adverse drug reactions. Early diagnose and early drug withdrawal are the keys to reduce adverse drug reactions. With cases' review and the summary in this article, we hope to improve clinicians' awareness about skin adverse drug reactions of heparin. We encourage clinicians to make routine follow-ups with pregnant women undergoing nadroparin calcium injection and evaluate their skin conditions.

## Figures and Tables

**Figure 1:** Illustrations of (a) erythemas at injection points on the abdomen and (b) urticaria-like reactions on the trunk in one individual.

**Table 1:** Clinical characteristics of localized and generalized skin adverse drug reactions in 6 pregnant women undergoing nadroparin calcium injection.

	Case 1	Case 2	Case 3	Case 4	Case 5	Case 6

Age	31	28	29	37	26	37
Incubation period	28	34	52	46	78	47
Total injection dose	39	46	65	63	104	68
Drug combination	Dydrogesterone	Dydrogesterone, estradiol	Dydrogesterone, euthyrox	Dydrogesterone	Dydrogesterone, estradiol	Dydrogesterone
Localized reactions at the injection point	Yes	Yes	Yes	Yes	Yes	Yes
Time of delayed reactions appeared	4	10	5	8	3	10
Manifestation of generalized reactions	Wheal	Wheal	Wheal	Wheal	Dermatographism	Wheal
Duration between appearances of localized and generalized reactions	7	5	2	6	1	11
Eosinophils count (×10^9^/L)	0.16	0.97	0.28	0.76	0.83	0.35
Treatments	Nadroparin calcium withdrawal, using desonide topical	Nadroparin calcium withdrawal, using calamine and mometasone ointment	Nadroparin calcium withdrawal, replacing with fondaparinux, using calamine and mometasone ointment	Nadroparin calcium withdrawal, replacing with enoxaparin, using calamine ointment, taking loratadine and chlorpheniramine	Nadroparin calcium withdrawal, taking loratadine and chlorpheniramine	Nadroparin calcium withdrawal, taking loratadine
Outcomes	All symptoms subsided in 2 weeks	All symptoms subsided in 4 weeks	All symptoms subsided in 3 weeks	All symptoms subsided in 2 weeks	All symptoms subsided in 5 weeks	All symptoms subsided in 3 weeks
Skin prick test	−	−	−	−	−	−
Skin patch test	−	−	−	−	−	−
Intradermal test	+	Declined	+	+	+	+

## Data Availability

The data used to support the findings of this study are available from the corresponding author upon request.

## References

[1] Hao C., Sun M., Wang H., Zhang L., Wang W. (2019). Low molecular weight heparins and their clinical applications. *Progress in molecular biology and translational science*.

[2] Hamulyák E. N., Scheres L. J., Marijnen M. C., Goddijn M., Middeldorp S. (2020). Aspirin or heparin or both for improving pregnancy outcomes in women with persistent antiphospholipid antibodies and recurrent pregnancy loss. *Cochrane Database of Systematic Reviews*.

[3] Hui C.-K., Yuen M.-F., Ng I. O.-L., Tsang K. W.-T., Fong G. C.-Y., Lai C.-L. (2001). Low molecular weight heparin-induced liver toxicity. *The Journal of Clinical Pharmacology*.

[4] Schindewolf M., Recke A., Zillikens D., Lindhoff-Last E., Ludwig R. J. (2017). Nadroparin carries a potentially high risk of inducing cutaneous delayed-type hypersensitivity responses. *Contact Dermatitis*.

[5] Polák P., Kaloudová Y., Krupicová H. (2020). Heparin-induced thrombocytopenia: a case report and literature overview. *Vnitrní Lékarství*.

[6] Brockow K., Garvey L. H., Aberer W. (2013). Skin test concentrations for systemically administered drugs - an ENDA/EAACI Drug Allergy Interest Group position paper. *Allergy*.

[7] Edwards I. R., Aronson J. K. (2000). Adverse drug reactions: definitions, diagnosis, and management. *The Lancet*.

[8] Schindewolf M., Gobst C., Kroll H. (2013). High incidence of heparin-induced allergic delayed-type hypersensitivity reactions in pregnancy. *The Journal of Allergy and Clinical Immunology*.

[9] Tramontana M., Hansel K., Bianchi L., Agostinelli D., Stingeni L. (2019). Skin tests in patients with delayed and immediate hypersensitivity to heparins: a case series. *Contact Dermatitis*.

[10] Ludwig R. J., Schindewolf M., Utikal J., Lindhoff-Last E., Boehncke W. H. (2006). Management of cutaneous type IV hypersensitivity reactions induced by heparin. *Thrombosis & Haemostasis*.

[11] Schindewolf M., Paulik M., Kroll H. (2018). Low incidence of heparin‐induced skin lesions in orthopedic surgery patients with low‐molecular‐weight heparins. *Clinical and Experimental Allergy*.

[12] Schindewolf M., Lindhoff-Last E., Ludwig R. J., Boehncke W.-H. (2012). Heparin-induced skin lesions. *The Lancet*.

[13] Arepally G. M., Padmanabhan A. (2021). Heparin-induced thrombocytopenia: a focus on thrombosis. *Arteriosclerosis, Thrombosis, and Vascular Biology*.

[14] Schindewolf M., Schwaner S., Wolter M. (2009). Incidence and causes of heparin-induced skin lesions. *Canadian Medical Association Journal*.

[15] Kim K. H., Lynfield Y. (2003). Enoxaparin-induced generalized exanthem. *Cutis*.

[16] Klos K., Spiewak R., Kruszewski J., Bant A. (2011). Cutaneous adverse drug reaction to heparins with hypereosinophilia and high IgE level. *Contact Dermatitis*.

[17] Trautmann A., Seitz C. S. (2009). Heparin allergy: delayed-type non-IgE-mediated allergic hypersensitivity to subcutaneous heparin injection. *Immunology and Allergy Clinics of North America*.

[18] Vu T. T., Gooderham M. (2017). Adverse drug reactions and cutaneous manifestations associated with anticoagulation. *Journal of Cutaneous Medicine and Surgery*.

[19] Bircher A., Itin P., Büchner S. (1994). Skin lesions, hypereosinophilia, and subcutaneous heparin. *The Lancet*.

[20] Staumont-Salle D., Dombrowicz D., Capron M., Delaporte E. (2006). Eosinophils and urticaria. *Clinical Reviews in Allergy and Immunology*.

